The article "Designing a Bioengine for Detection and Analysis of Base String on an Affected Sequence in High-Concentration Regions" was retracted in 2021. Reasons: plagiarism; overlap with other authors' work.

# Designing a Bioengine for Detection and Analysis of Base String on an Affected Sequence in High-Concentration Regions

**DOI:** 10.1155/2013/372646

**Published:** 2013-08-13

**Authors:** Debnath Bhattacharyya, Bijoy Kumar Mandal, Tai-hoon Kim

**Affiliations:** ^1^Department of Computer Science & Engineering, Faculty of Engineering and Technology, NSHM Knowledge Campus, Durgapur 713212, India; ^2^Department of Convergence Security, Sungshin Women's University, 249-1, Dongseon-dong 3-ga, Seoul 136-742, Republic of Korea

## Abstract

We design an Algorithm for bioengine. As a program are enable optimal alignments searching between two sequences, the host sequence (normal plant) as well as query sequence (virus). Searching for homologues has become a routine operation of biological sequences in 4 × 4 combination with different subsequence (word size). This program takes the advantage of the high degree of homology between such sequences to construct an alignment of the matching regions. There is a main aim which is to detect the overlapping reading frames. This program also enables to find out the highly infected colones selection highest matching region with minimum gap or mismatch zones and unique virus colones matches. This is a small, portable, interactive, front-end program intended to be used to find out the regions of matching between host sequence and query subsequences. All the operations are carried out in fraction of seconds, depending on the required task and on the sequence length.

## 1. Introduction

It is known that viroids are the smallest replicating pathogenic agents (see [1] for relevant references), which is entirely composed of RNA with genome sizes in the range of 330–380 nucleotides [2], that is 10 times smaller than the smallest bacteriophage of *Escherichia coli* [3]. It is also known that they infect a wide variety of plants and produce severe disease symptoms in many plants [4–12], but there is no evidence for the existence of a protective protein coat for viroids. The molecular mechanisms by which viroids replicate and interact with their hosts are not yet understood. In its most severe form, the disease [5, 6] caused by potato spindle tuber viroid (PSTV) causes general stunting of potato plant growth, deformity of the upper foliage, and production of disfigured potatoes [5]. Mild strains of PSTV which produce barely detectable symptoms have also been isolated [7]. Furthermore, plants infected with mild strains are somehow protected from developing symptoms following subsequent inoculation with severe strains [8, 9]. The sequence of the 247 nucleotide residues of the single strand circular RNA of avocado sunblotch viroid (ASBV) was determined using partial enzymes cleavage methods on overlapping viroid fragments obtained by partial ribonucleic digestion followed by ^32^p-labelling *in vitro* at their 5′-ends. ASBV is much smaller than potato spindle tuber viroid (PSTV; 359 residues) and chrysanthemum stunt viroid (CSV; 356 residues). The sequences of the viroid progeny and the cloned DNA were identical. *In vitro* mutagenesis of infectious PSTV cDNAs will allow systematic investigation of the role of specific sequences in viroid replication and pathogenesis [10]. A complex of considerable stability is possible between the 5′-end of U1 RNA and a specific nucleotide sequence of the potato spindle tuber viroid complement. Small nuclear RNAs (snRNAs) that are associated with ribonucleoprotein particles are believed by some to be involved in the processing of the primary transcription products of split genes. The 5′-end of one such RNA, U1, has been shown to exhibit complementarity with the ends of introns, and it is believed that this affords a mechanism ensuring correct excision of the intron sequences and accurate joining of the coding sequences [11]. The invention provides a novel retroviral packaging system, in which retroviral packaging constructs and packageable vector transcripts are produced from high-expression plasmids by replicating in a human's cell via the enzyme reverse transcriptase to produce DNA from its RNA genome. Retroviruses are enveloped viruses that belong to the viral family retroviridae. High titers of recombinant retrovirus are produced in infected cells. The methods of the invention include the use of the novel retroviral constructs to transduce primary human cells, including T cells and human hematopoietic stem cells, with foreign genes by cocultivation at high efficiencies. The invention is useful for the rapid production of high viral supernatants, and to transduce with high-efficiency cells that are refractory to transduction by conventional means [12].

## 2. Basis of the Algorithm

There are four issues which are focused mainly to provide for detection of a fixed base string on an affected sequence.

### 2.1. Similarity

To define similarity, perhaps it is useful to first introduce the notion of “distance” between two strings. The distance between two strings is zero if they are exactly the same. The distance between two strings increases if they get more dissimilar. One way of defining distance between two strings is to look at the amount of change they needed to do to one to obtain the other. They could go on to introduce other changes, insert, and delete. Insert “happens” when they inserted some letter into the sequence (at some position), and delete happens when they deleted some letter at some position.

### 2.2. Edit Distance

This is defined as the minimum number of changes to be performed on one sequence to make it exactly the same as another.

### 2.3. Alignment of Sequence

For every two sequences, there are huge permutations of possible alignments (cubic in the length of sequences). Alignment procedure itself can be visualized as a series of insert, delete operations. 

### 2.4. Scoring Function

A scoring function determines this notion of goodness of alignment. They could compute the distance between alignments in such a way that the cost of a match is 0 (when the sequence on top and below has the same *i*th character). Cost of a mismatch is that they could choose different scoring schemes. Another sample scoring scheme could give lesser weights for replacement of A by T, and G by C (and vice versa) as against replacement of A by G or the others. Domain knowledge is used while determining scoring schemes.

## 3. Designing of the Algorithm

There are basic steps that constitute the whole process of analysis for high-concentration regions (HCR) detection of a fixed base string on an affected sequence and those steps are as follows.

### 3.1. Match Occurs in the following Way

 
*Q*[*i*] = *H*[*j*] to *H*[*m* − *L* + 1].
 As for example, *Q*[1] = *H*[1] first match found.
 Next *Q*[2] match with *H*[1] to *H*[*m* − *L* + 1].
 This process will continue at the end of query sequence. This process is repeated at the end of query sequence, until all possible matches are found.
 Match found then *Q*[*i*] = *H*[*j*].

### 3.2. Analysis of Matching Method

 The analysis of matching method is done in four different parts.

#### 3.2.1. Consider a DNA Sequence and Their Related Changes

 1 2 3 4 5 6 7 8 9 10 11 12…………*n*
 DNA CG G A A C T A A A C T C …………*n*_*n*_
 RNA CG G A A C U A A A C U C …………*n*_*n*_
 cDNA G C C T T G A T T T G A G …………*n*_*n*_
 cRNA GC C U U G A U U U G A G …………*n*_*n*_,

where, *n* is the number of bases in the nucleotide sequence.

*n*_*n*_ is the *n*th (i.e., last) base (A/T/G/C) in host and query genome sequences, which consist of bases A, T, G, and C (note that T is replaced with U in the case of the RNA). This example is applicable both in host and query sequences, and *n* is the length of the sequence in both cases, but they are the same or do not depend on user.

#### 3.2.2. Generating the Query Subsequence from Input Sequence

They broke the host and query sequence into user requirement subsequences length for easy implementation of Figure 1.

From Figure 1 pictorial representation, it is clear that for *i*th subsequence *W*_*i*_ (called colons): *i* is the starting position of the subsequence and *j* = (*i* − 1) + *L* is end position of the subsequence, where *L* is the subsequence length (word size). For example, if word size is 4, then:

For

*W*_1_ starting position (*i*) = 1 and (end position) *j* = (1 − 1) + 4 = 4,
*W*_2_ starting position (*i*) = 2 and (end position) *j* = (2 − 1) + 4 = 5 and
*W*_3_ starting position (*i*) = 3 and (end position) *j* = (3 − 1) + 4 = 6 and so on.

The clones with word size less than 3 (three) has no importance in matching context and hence we considered the clones with word size in the range: 3 ≤ *L* ≤ *n*.

Therefore, ranges for *i* and *j* are as 3 ≤ *i* ≤ *n* − *L* + 1 and *L* + 1 ≤ *j* ≤ *n*, respectively.

The subsequence generation time, both in host and query sequences cases, at the end (subsequence  length − 1) number of nucleotide base pair (a, t, g, and c) remains as it is. This is the reason why probability of infection decreases. To solve this problem, we have to find the result in reverse order.

The host sequence is defined by *H* and query sequence is defined by *Q*; each of the sequences must have the same or different lengths.

So, we could write

*H* = ATGCTAGCAGTAGACGATAGC………*n*,  *n* > 0 and *T* = TGCAGTAGCAGATGAC…………*m*,  *m* > 0, where *n* and *m* are the length of host and query sequences.

After subsequence division, they could get the result as follows.

So, they could rewrite *H*[*i*] = *H*[1]*H*[2]………*H*[*n* − *L* + 1],  1 ≤ *i* ≤ *n* − *L* + 1 and *Q*[*j*] = *Q*[1]  *Q*[2]………*Q*[*m* − *L* + 1],  1 ≤ *j* ≤ *m* − *L* + 1.

If the subsequence length or word size is *L* (3 < *L* ≤ *n* − *L* + 1).

If the number of subsequence is *S*, the total number of subsequences is generated in case that host sequence is 1 ≤ *S* ≤ *n* − *L* + 1 and case that query sequences is 1 ≤ *S* ≤ *m* − *L* + 1.

This subsequence method is required to reduce the complexity of the program execution.

#### 3.2.3. Matching between Host and Query Sequence

Let us look for matches in between Host sequence and Query sequence in Table 1. 

Here, host sequence is the virus sequence and Query sequence is the Tomato chloroplast,… and so forth, complete genome sequence of the Tomato plant and Root sequence.

16 possible matches may occur, and matches found are shown in the following:

 DNA versus DNA
 DNA versus RNA
 DNA versus cDNA
 DNA versus cRNA
 RNA versus DNA
 RNA versus RNA
 RNA versus cDNA
 RNA versus cRNA
 cDNA versus DNA
 cDNA versus RNA
 cDNA versus cDNA
 cDNA versus cRNA
 cRNA versus DNA
 cRNA versus RNA
 cRNA versus cDNA
 cRNA versus cRNA.

In these cases, the value of *i* is incremented by *i* = no. of unmatched character + no. of substring match × 3; similarly *j* is incremented by this same procedure.

Otherwise *Q*[*i*] ≠ *H*[*j*]; that is, unmatched occurs, the value of *i* and *j* is incremented by one.

At the end, we could get the result as Table 2.

Host and Query sequence infections are calculated by *|*NBM*|*/*||*TL*|* where NBM is the total no of base pair match, which is equivalent to total number word match multiplied by word size, is divided by length of host sequence in case of virus infection, length of query sequence in case of plant infection.

#### 3.2.4. Threshold Value

Proving this hypothesis, we have considered a threshold value, on this threshold value we can take the decision as described as follows.

- Infectivity “HIGH” means that the virus is highly infectious on target sequence; that is, chloroplast of the tomato plant is infected by PSTVd virus from head to tail. In this situation, the infection between the source (PSTVd) and the target sequence (tomato chloroplast) is very high.
- Infectivity “NEGLIGIBLE” means that the virus is infected on target sequence; that is, chloroplast of the tomato plant is infected by PSTVd virus from head to tail are not infected. In this situation, the infection between the source (PSTVd) and the target sequence (tomato chloroplast) is infected, but it is not harmful.
- Infectivity “LOW” means the virus infection is found, but not so called infectious on target sequence; that is, chloroplast of the tomato plant is infected by PSTVd virus from head to tail are not infected. In this situation, the infection between the source (PSTVd) and the target sequence (tomato chloroplast) is noninfectious.

## 4. Experimental Data

### 4.1. Matches between Host Sequence and Query Sequence

This aspect is given in Figure 2.

### 4.2. Alignment Demo

The matter of alignment is shown in Figure 3.

### 4.3. Pictorial Representation Shows That Match Region

The pictorial representation of matched region is shown in Table 3 (word size 3).

### 4.4. Highest Matching Word

The highest matched word is given in Table 4.

## 5. Project Spectrum

We have the following:

- A base program to detect the HCRs in a target sequence for a given viral sequence.
- A method to locate the start and end positions of infection and isolate the infected regions.
- A method to identify the longest infected region or the largest HCR.
- An extension to allow all 4 possible transforms of the viral sequence (i.e., DNA, RNA, cDNA, and cRNA).
- An extension to allow scanning of all possible transforms of the normal plant (target) sequence, that is, DNA, RNA, cDNA, and cRNA. A total of 4×4 scan orientations.
- An extension to identify successive regions of *Edit Distance* = 1.
- An extension to detect and report all such extrapolated infection regions and locate the largest of them.

## 6. Architecture of Process

The required architecture for the whole process is shown in Figure 4.

### 6.1. Inputs

- The Inputs Taken are
  - normal plant sequence:
    - a steam of DNA bases in FASTA format, that is, a text file containing an DNA sequence.
    - limitations: none.
  - viral sequence:
    - a steam of RNA bases in fasta format, that is, a text file containing an RNA sequence.
    - limitations: size of file should be less than 400 Kbytes.   

### 6.2. Codon Generator

Codon Generator is shown in Figure 5.

### 6.3. Codon Tree

The structure of codon tree is given in Figure 6.

### 6.4. Transforms

The process of transformation is shown in Figure 7.

### 6.5. Sequence Analyzer

The process of sequence analyzer is given in Figure 8.

## 7. Complexity

The algorithm uses an *M*-array tree to structure the input sequence and then allows the target to “pour through” the root and fit in place. Thus, the target sequence looks at a match, rather than the other way round. Here, *M* = 5 so the time complexity of the program is

 O(*n*_1_  log⁡_*M*_ O(*n*_1_  log⁡_5_ *n*_2_)*n*_2_)
 O  (*n*_1_  log⁡_5_ *n*_2_)
 
*n*_1_: size of viral sequence
 
*n*_2_: size of plant sequence.

## 8. Analysis

A comparison of a variant of the same program, using the strcmp() library function yielded the following timings. This is tabulated in Table 5.

## 9. Performance

The program was tested with real inputs and the time spent is tabulated in Table 6.

## 10. Conclusion

This algorithm shows that virus and normal plant interaction was found only in between virus RNA with normal plant cDNA and RNA stand only. The virus and plant interaction was found only in normal in nature, no such other orientation is applicable. The colon size varies from 3 to 9. The lower the subsequence size, the higher the interaction rate. This algorithm also can apply on any type of virus and any type of normal plant genome sequences. In future, an attempt will be made to apply this software in real-life example such as Potato Spindle Tuber Viroid infected only chloroplast of the Tomato plant not in their root.

## Figures and Tables

**Figure 1:** 

**Figure 2:** Matches between Host Sequence and Query Sequence.

**Figure 3:** Alignment demo.

**Figure 4:** Architecture of process.

**Figure 5:** Codon generator.

**Figure 6:** Codon tree.

**Figure 7:** Process of transformation.

**Figure 8:** Sequence analyzer.

**Table 1:** 

Source sequence Target sequence	
DNA *→* DNA	
RNA *→* RNA	
cDNA *→* cDNA	
cRNA *→* cRNA	

**Table 2:** 

	*H*[1] *H*[5]*H*[6] ………………*H*[*n* − *L* + 1]
Source sequence	*S*[*i*] : CGG C U AAAC………………….*n*
Target sequence	*T*[*i*] : CG G A A C U A A A C U C ………*m*
	*T*[1] *T*[4]*T*[5]………….*T*[*m* − *L* + 1]
Total word match = 3	

**Table 3:** Pictorial representation for showing the match region.

Position	Match position	Total base pair match	Gap	Highest match position without gap	Highest match position with gap
1st position	1–6 (1–3 and 4–6)	6	0		
2nd position	8–10	3	1		
3rd position	12–14	3	1		
4th position	17–22	6	2		
5th position	25–36	12	2	25–33	
6th position	38–39	3	1		25–39

**Table 4:** Highest matching word.

Words/colones	Repeat numbers
ATG	3
TTT	5
TAT	1
TGC	1

**Table 5:** Analysis of present algorithm.

Target input with fixed base sequence, 349 bytes	Time with strcmp()	Time with this Algorithm
200 KB	200 seconds	25 milliseconds
1 MB	7 minutes	456 milliseconds
1.5 MB	15 minutes	1-2 second (s)
>2 MB	The computer hanged	~15 seconds

**Table 6:** Performance of viruses of different size.

Virus (in KB)	Plant (in KB)	Time taken
<400 bytes	<5	~0.5 milliseconds
500–1024 bytes	<5	~0.5 milliseconds
1–5	<100	~90 milliseconds
1–5	200–1024	~400 milliseconds
10–100	1024–5 MB	~1–4 seconds
10–100	5–7 MB	~5–10 seconds
100–300	~10	~15–20 seconds
